The article "Modified Prehospital Acute Stroke Severity (mPASS) Scale to Predict Emergent Large Arterial Occlusion" was retracted in 2024. Reasons: signs of a paper mill; suspected computer-generated content; unreliable results or conclusions; concerns about the data.

# Modified Prehospital Acute Stroke Severity (mPASS) Scale to Predict Emergent Large Arterial Occlusion

**DOI:** 10.1155/2021/5568696

**Published:** 2021-07-19

**Authors:** Xiaoli Si, Jie Ruan, Lingfei Li, Shan Lu, Huan Huang, Wenqing Xia, Keqin Liu, Tianwen Chen, Lin Jiang, Congguo Yin

**Affiliations:** ^1^Department of Neurology, Second Affiliated Hospital, College of Medicine, Zhejiang University, Hangzhou, Zhejiang, China; ^2^Department of Neurology, Hangzhou Geriatric Hospital, Hangzhou, China; ^3^Department of Neurology, Affiliated Hangzhou First People's Hospital, Zhejiang University School of Medicine, Hangzhou, China

## Abstract

**Introduction:**

To date, identifying emergent large vessel occlusion (ELVO) patients in the prehospital stage is important but still challenging. In this present study, we aimed to design a modified prehospital acute stroke severity (mPASS) scale to identify ELVO patients and compared the scale to the PASS scale which has been published.

**Methods:**

We retrospectively evaluated a consecutive cohort of acute ischemic stroke (AIS) in our stroke unit who visited the emergercy department. These patients underwent CT angiography (CTA), MR angiography (MRA), or digital subtraction angiography (DSA) at admission. The mPASS scale was calculated based on the National Institutes of Health Stroke Scale (NIHSS) items retrospectively, including the level of consciousness commands, gaze, arm weakness, and aphasia/dysarthria. Receiver operating characteristic (ROC) analysis was used to obtain the area under the curve (AUC) of the mPASS scale, NIHSS, and PASS scale. *U*-statistics was used to compare the AUC of the mPASS scale to the NIHSS and PASS scale.

**Results:**

A total of 382 AIS patients were enrolled. The AUC and specificity of the mPASS scale (0.92, 84.4) were all higher than those of the PASS scale. Cortical symptoms such as gaze palsy and consciousness disorder were more specific indicators for ELVO than motor deficits.

**Conclusions:**

The mPASS scale had a better discrimination for identifying ELVO than the PASS scale in our retrospective cohort. It might predict ELVO in an effective and simple way for paramedics in the prehospital triage stage or emergency stage. Moreover, cortical symptoms might have relatively high specificities to predict ELVO on their own.

## 1. Introduction

Reperfusion with the intravenous tissue plasminogen activator (recombinant tissue-type plasminogen activator (rt-PA)) and endovascular therapy (EVT) improve outcomes in acute ischemic stroke (AIS) patients [1]. Both treatment efficiencies are highly time dependent [2]. Intravenous thrombolysis can be administered in Primary Stroke Centers (PSCs) while endovascular treatment can only be administered in EVT-capable centers in Comprehensive Stroke Centers (CSCs) [3]. Several recent studies have demonstrated that patients may have a better outcome by shortening the delay to EVT. Therefore, a simple and accurate assessment for paramedics to precisely identify emergent large vessel occlusion (ELVO) in the setting of prehospital triage stage or emergency stage is urgent.

The article "Modified Prehospital Acute Stroke Severity (mPASS) Scale to Predict Emergent Large Arterial Occlusion" was retracted in 2024. Reasons: signs of a paper mill; suspected computer-generated content; unreliable results or conclusions; concerns about the data.

Computed tomography angiography (CTA), magnetic resonance angiography (MRA), or digital subtraction angiography (DSA) allow a rapid assessment of the vessel status in AIS. However, they are not broadly available 24 hours per day, particularly for PSCs with imaging resources limited [4]. Thus, surrogate clinic markers of vessel occlusion will be helpful. The National Institutes of Health Stroke Scale (NIHSS) has a relatively strong relationship between neurological deficit and vessel status [5]. However, it is complex for emergency assessment and necessitating regular training for primary paramedics.

There have been several prehospital stroke scales to identify patients experiencing ELVO [6–9]. Among them, the Prehospital Acute Severity Scale (PASS) simplifies the parameters and has been shown to improve the predictive capability of ELVO when compared to other reported scales [10]. The PASS scale (level of consciousness (LOC) questions, which combined both assessments of language and consciousness (scored 0–1), gaze palsy and/or deviation (0–1), and arm weakness (scored 0–1)) is derived from the NIHSS. The PASS scale score ≥ 2 predicts ELVO. However, patients with basal ganglia infarction (non-emergent large vessel occlusion) may get a PASS score = 2, if they have slurred speech and arm weakness. Therefore, it is unsuitable to evaluate the level of consciousness (LOC) through LOC questions in the PASS scale. In this present study, we replaced the item “LOC questions” by the item “LOC commands—open/close eyes, grip, and release non-paretic hand” to evaluate LOC in our scale. And we add the item “aphasia” separately. However, in emergency evaluation, paramedics could not accurately distinguish speech ambiguity as aphasia or dysarthria and cortical symptoms of some patients with right hemisphere infarction could also be manifested as dysarthria. Therefore, aphasia and dysarthria are both included in language evaluation indicators. Here, we developed a new scale—the modified Prehospital Acute Stroke Severity (mPASS) Scale, which is derived from the PASS scale. We posit that the modification of the PASS scale might increase the predictive ability of ELVO. Then, we retrospectively evaluated whether the mPASS scale could achieve a better predictive performance than the PASS scale for identifying ELVO.

The article "Modified Prehospital Acute Stroke Severity (mPASS) Scale to Predict Emergent Large Arterial Occlusion" was retracted in 2024. Reasons: signs of a paper mill; suspected computer-generated content; unreliable results or conclusions; concerns about the data.

## 2. Subjects and Methods

We retrospectively reviewed a historical cohort of 720 patients who visited the emergency room from January 2016 to January 2018 in Hangzhou First People's Hospital, Zhejiang University. We enrolled patients who (1) were clinically suspected of AIS (symptom onset ≤ 24 hours, including patients who have intracerebral hemorrhage (ICH) or with a final nonvascular diagnosis like status epilepticus, syncope, metabolic disturbance, and other reasons) at emergency, (2) were examined by 2 experienced stroke neurologists and assessed with the NIHSS at the emergency room (the assessment of the NIHSS was written on sheets detailed to each parameter), (3) were AIS patients confirmed by magnetic resonance imaging (MRI) diffusion-weighted imaging (DWI) at admission, and (4) were ELVO patients confirmed by CTA, MRA, or DSA at admission. Participants' baseline demographic (age, gender, and smoking), clinical characteristics (diabetes, hyperlipidemia, hypertension, and atrial fibrillation), laboratory data (serum glucose at admission, low-density lipoprotein, and homocysteine), and images were recorded.

The mPASS was calculated based on NIHSS retrospectively by 2 experienced neurologists. This scale assessed 4 parameters: (1) LOC commands—open/close eyes, grip, and release the nonparetic hand (scored 0 and 2); (2) gaze (scored 0 and 2); (3) arm weakness (scored 0 and 1); and (4) aphasia/dysarthria (scored 0 and 1) (Table 1).

ELVO is defined as occlusion of the internal carotid artery (ICA), anterior cerebral artery (ACA), horizontal segment (M1), and insula segment (M2) of middle cerebral artery (MCA), posterior cerebral artery (PCA), basilar artery (BA), and vertebral artery (VA). Two experienced neurologists blinded to patients' information assessed the occlusion on CTA, MRA, or DSA with rater discrepancies settled by consensus. Patients with inconclusive or missing information on NIHSS or were not eligible for imaging assessment were excluded. The flowchart of the study population is shown in Figure 1. This study was approved by the ethics committee of the Affiliated Hangzhou First People's Hospital, Zhejiang University School of Medicine, and written consent was obtained from each participant.

### 2.1. Statistical Analysis

Patients were divided into the AIS-ELVO group and AIS-non-ELVO (NELVO) group. Data were entered into Microsoft Excel, and statistical analyses were performed with Statistical Package for the Social Sciences 18.0 (IBM, Chicago, IL, USA). Statistical plots were generated using GraphPad Prism 7.0a (GraphPad Inc., San Diego, CA, USA). Categorical or binary datum was summarized by proportion (*n*, %), clinical characteristics were presented as mean ± standard deviation (mean ± SD) and as median (interquartile range (IQR)). The Kolmogorov-Smirnov test was used to determine the normality of the distribution of the variables. Demographic data, clinical variables, and scale scores were compared using independent *t*-tests for normally distributed continuous variables, and Mann–Whitney *U* test and Kruskal-Wallis *H* test for continuous variables that were not normally distributed. Receiver operating curves (ROC) and areas under receiver operating curve (AUC) were calculated as measures of predictive ability for ELVO among AIS patients (ELVO and AIS-ELVO) of the mPASS scale, PASS scale, and NIHSS and for different items of the mPASS scale. ROC-derived optimal cutoff was determined at the maximal Youden index. Cross tables for different cutoff values of the mPASS scale were used to evaluate sensitivity, specificity, positive predictive value (PPV), and negative predictive value (NPV). A value with *p* < 0.05 was regarded as statistically significant.

The article "Modified Prehospital Acute Stroke Severity (mPASS) Scale to Predict Emergent Large Arterial Occlusion" was retracted in 2024. Reasons: signs of a paper mill; suspected computer-generated content; unreliable results or conclusions; concerns about the data.

## 3. Results

Totally, we screened 720 patients in our stroke unit from January 2016 to January 2018. Finally, 382 AIS patients were included. Figure 1 summarized the flowchart of the study population. In the ELVO group, the mean age was 70.3 ± 11.2 years, males were 111 (60.7%), median time between symptom onset and assessment was 4.7 ± 4.0 hours, and median NIHSS score was 17.2 ± 8.0. In the NELVO group, the mean age was 71.0 ± 11.2 years, males were 118 (59.3%), median time between symptom onset and assessment was 9.7 ± 5.1 hours, and median NIHSS score was 4.6 ± 4.6. The AUC of the mPASS scale to predict ELVO from AIS (ELVO and AIS-NELVO patients) was 0.917. The highest Youden index was 0.751, which was achieved for a mPASS score ≥ 3, with sensitivity, specificity, PPV, and NPV of 0.907, 0.844, 0.843, and 0.908, respectively. The AUC of the PASS scale was 0.878. The highest Youden index was 0.785, which was achieved for a PASS score ≥ 2, with sensitivity, specificity, PPV, and NPV of 0.945, 0.839, 0.844, and 0.944, respectively. The AUC of the NIHSS was 0.944. The highest Youden index was 0.778, which was achieved for a NIHSS score ≥ 9, with sensitivity, specificity, PPV, and NPV of 0.929, 0.849, 0.841, and 0.923, respectively. The AUC of the mPASS scale was significantly higher than that of the PASS scale (*p* < 0.05) (Figure 2, Table 2).

Figure 3 showed that the strongest predictor of ELVO through mPASS scale's four parameters was gaze palsy and/or deviation, with AUC = 0.788 (95% confidence interval (CI) 0.741-0.836), sensitivity 73.8%, and specificity 83.9%. The second strongest predictor was LOC command, with AUC = 0.717 (95% CI, 0.665-0.770), sensitivity 59.6%, and specificity 83.9%. Then comes aphasia/dysarthria which showed AUC = 0.713 (95% CI, 0.661-0.765), sensitivity 98.9%, and specificity 43.7%. The last is arm weakness, which showed AUC = 0.639 (95% CI, 0.584-0.695), sensitivity 96.7%, and specificity 31.2%. The ELVO group had a higher percentage of LOC command and gaze palsy than the AIS-NELVO group (Mann–Whitney *U* test, *p* < 0.001). ACI had a higher percentage of gaze palsy (Mann–Whitney *U* test, *p* < 0.001), and PCI had a higher percentage of consciousness disorder (Mann–Whitney *U* test, *p* = 0.003). Detailed vessel occlusion types were ACA 2 (1.1%), ICA 54 (29.5%), MCA 95 (51.9%), PCA 2 (1.1%), BA 29 (15.8%), and VA 1 (0.5%). We ran a separate analysis using only ICA/M1 occlusions as the ELVO definition. The AUC of the mPASS scale to predict ELVO from AIS (ELVO and AIS-NELVO patients) was 0.926. The highest Youden index was 0.763, which was achieved for mPASS score ≥ 3, with sensitivity, specificity, PPV, and NPV of 0.919, 0.844, 0.815, and 0.933, respectively. The AUC of the PASS scale was 0.883. The highest Youden index was 0.785, which was achieved for PASS score ≥ 2, with sensitivity, specificity, PPV, and NPV of 0.946, 0.839, 0.815, and 0.954, respectively. The AUC of the NIHSS was 0.941. The highest Youden index was 0.782, which was achieved for a NIHSS score ≥ 9, with sensitivity, specificity, PPV, and NPV of 0.939, 0.849, 0.822, and 0.944, respectively (in supplementary materials).

The article "Modified Prehospital Acute Stroke Severity (mPASS) Scale to Predict Emergent Large Arterial Occlusion" was retracted in 2024. Reasons: signs of a paper mill; suspected computer-generated content; unreliable results or conclusions; concerns about the data.

## 4. Discussion

The NIHSS has demonstrated to be predictive of ELVO, but is difficult and time-consuming for PSC paramedics who are inexperienced in performing assessment. Moreover, right hemispheric ELVO may present mild to moderate symptoms underrepresented with the NIHSS which would be ignored. Currently, a European group has designed and demonstrated the PASS scale as a simple tool that highly predicts ELVO emergency. The current study indicates that our novel mPASS in retrospective cohort had a good discrimination ability and could be an easily memorized tool to identify ELVO, as the AUC of the mPASS scale showed a higher predictive value compared with the NIHSS and PASS scale. Atherosclerotic intracranial stenosis is found commonly among stroke patients of Asian, Black, and Hispanic ancestry [11], especially in China [12]. Thus, the mPASS scale would be a useful and necessary tool to detect ELVO patients, especially for Asian patients.

There are several advantages of the mPASS scale over existing scales. First, parameters in the mPASS are easily observed and objective to evaluate. LOC commands are objective and could be separated with evaluation of aphasia/dysarthria which the PASS scale ignored [10]. Gaze palsy can be easily observed by paramedics in emergency conditions rather than neglect or field of vision in RACE, FAST-ED, and VAN scales [13, 14]. Second, the different forms of the PASS, 3ISS, LAMS, and mPASS scales give a higher weight to cortical symptoms (consciousness disorder 0/2, gaze palsy, and/or deviation 0/2) rather than motor symptoms (arm weakness 0/1), which are typical signs of ELVO, because motor symptoms can also occur in lacunar stroke and may not be good indicators for ELVO. This study also indicated that the strongest predictor was cortical symptoms (consciousness disorder and gaze palsy and/or deviation). Recently, gaze palsy and/or deviation has been the only parameter in an ELVO screen as an ideal prehospital scale [11]. Thus, we may further design a simpler and faster scale which just focuses on cortical symptoms and validates prospectively in the field by trained paramedics prehospital in the future.

The article "Modified Prehospital Acute Stroke Severity (mPASS) Scale to Predict Emergent Large Arterial Occlusion" was retracted in 2024. Reasons: signs of a paper mill; suspected computer-generated content; unreliable results or conclusions; concerns about the data.

Our study has several limitations. First, this model was made from a single retrospective cohort. Perspective and large multicenter data would be more believable and compelling. Second, as a global scale with a limited range (0 to 6), the mPASS scale is insensitive to small differences between patients and to small changes in clinical status for individual patients. However, the complexity of the NIHSS scale is responsible for its infrequent use in clinical routine. In contrast, the mPASS scale is relatively more simple and faster to apply. Moreover, the mPASS score in ACI was higher than that in PCI; however, NIHSS score was higher in PCI than ACI. The accuracy of the mPASS scale in PCI needs further investigation and improvement.

## 5. Conclusion

In summary, the mPASS scale might be an easily memorized and effective tool to identify AIS with high likelihood of ELVO. The mPASS scale might achieve a better predictive performance than the PASS scale for identifying ELVO. Additional studies concerning utility and accuracy of the mPASS scale in prehospital setting and its ability to predict stroke outcome are warranted, which may change destination triage decisions and transfer appropriate patients to a CSC more quickly.

## Figures and Tables

**Figure 1:** Flowchart of the study population. NIHSS: National Institutes of Health Stroke Scale; CTA: computed tomography angiography; MRA: magnetic resonance angiography; DSA: digital subtraction angiography; AIS: acute ischemic stroke; N-AIS: nonacute ischemic stroke; ELVO: emergent large vessel occlusion; NELVO: non-emergent large vessel occlusion; ICH: intracerebral hemorrhage.

The article "Modified Prehospital Acute Stroke Severity (mPASS) Scale to Predict Emergent Large Arterial Occlusion" was retracted in 2024. Reasons: signs of a paper mill; suspected computer-generated content; unreliable results or conclusions; concerns about the data.

**Figure 2:** Discrimination and calibration analysis: mPASS scale showed AUC 0.917, sensitivity 90.7%, and specificity 84.4%; the PASS scale showed AUC 0.878, sensitivity 94.5%, and specificity 83.9%; the NIHSS showed AUC 0.944, sensitivity 92.9%, and specificity 84.9%.

**Figure 3:** Discrimination and calibration analysis: level of consciousness showed AUC = 0.717, sensitivity 56.9%, and specificity 83.9%; gaze palsy and/or deviation showed AUC = 0.788, sensitivity 73.8%, and specificity 83.9%; aphasia/dysarthria showed AUC = 0.713, sensitivity 98.9%, and specificity 43.7%; arm weakness showed AUC = 0.639, sensitivity 96.7%, and specificity 31.2%.

**Table 1:** The mPASS scale and its correspondence to the PASS scale and NIHSS.

Item	mPASS	NIHSS
LOC commands		
Both correct	0	0
One correct	1	1
Neither correct	2	2
Gaze		
Normal	0	0
Partial deviation	1	1
Forced deviation	2	2
Arm weakness		
No drift/drift but does not hit bed	0	0–1
Drift and hit bed/no effort against gravity/no movement	1	2–4
Aphasia/dysarthria		
Normal	0	0
Aphasia and/or dysarthria	1	1–3/1–2

LOC: level of consciousness; mPASS: modified Prehospital Acute Stroke Severity; NIHSS: National Institutes of Health Stroke Scale.

**Table 2:** Sensitivity, specificity, PPV, NPV, and overall accuracy of different scales.

Scale	AUC	95% CI	Sensitivity (%)	Specificity (%)	PPV (%)	NPV (%)	Youden (%)	Accuracy (%)
mPASS ≥ 3	0.917	0.889–0.944	90.7	84.4	84.3	90.8	75.1	87.4
Pass ≥ 2	0.878	0.833–0.916	94.5	83.9	84.4	94.4	78.5	89.0
NIHSS ≥ 9	0.944	0.921–0.967	92.9	84.9	84.1	92.3	77.8	88.7

mPASS: modified Prehospital Acute Stroke Severity; PASS: Prehospital Acute Stroke Severity; NIHSS: National Institutes of Health Stroke Scale; AUC: area under the curve; CI: confidence interval; PPV: positive predictive value; NPV: negative predictive value.

## Data Availability

We confirm that our article contains a data availability statement. We confirm that we have included a citation for available data in our reference section. The data that support the findings of this study are openly available.

## Supplementary Materials

Supplementary Materials We ran a separate analysis using only ICA/M1 occlusions as the ELVO definition. Tables 3, 4, and 5 are sensitivity, specificity, PPV, NPV, and overall accuracy of different scales. Figure 4: discrimination and calibration analysis: the mPASS showed AUC 0.917, sensitivity 90.7%, and specificity 84.4%; the PASS showed AUC 0.876, sensitivity 92.6%, and specificity 83.9%; the NIHSS showed AUC 0.935, sensitivity 88.9%, and specificity 89.9%(AIS-ICA/NELVO). Figure 5: discrimination and calibration analysis: the mPASS showed AUC 0.931, sensitivity 92.6%, and specificity 84.4%; the PASS showed AUC 0.887, sensitivity 95.8%, and specificity 83.9%; the NIHSS showed AUC 0.944, sensitivity 93.7%, and specificity 84.9% (AIS-MCA-M1/NELVO). Figure 6: discrimination and calibration analysis: the mPASS showed AUC 0.926, sensitivity 91.9%, and specificity 84.4%; the PASS showed AUC 0.883, sensitivity 94.6%, and specificity 83.9%; the NIHSS showed AUC 0.941, sensitivity 93.3%, and specificity 84.9% (AIS − ICA + MCA − M1/NELVO).
